This article has been retracted.

# Astakine 2—the Dark Knight Linking Melatonin to Circadian Regulation in Crustaceans

**DOI:** 10.1371/journal.pgen.1003361

**Published:** 2013-03-21

**Authors:** Apiruck Watthanasurorot, Netnapa Saelee, Amornrat Phongdara, Sittiruk Roytrakul, Pikul Jiravanichpaisal, Kenneth Söderhäll, Irene Söderhäll

**Affiliations:** 1 Department of Comparative Physiology, Uppsala University, Uppsala, Sweden; 2 Center for Genomics and Bioinformatics Research, Faculty of Science, Prince of Songkla University, Songkhla, Thailand; 3 Proteomics Research Laboratory, Genome Institute, National Center for Genetic Engineering and Biotechnology (BIOTEC), NSTDA, Pathumthani, Thailand; 4 Aquatic Molecular Genetics and Biotechnology Laboratory, National Center for Genetic Engineering and Biotechnology (BIOTEC), NSTDA, Pathumthani, Thailand; Wellesley College, United States of America

## Abstract

Daily, circadian rhythms influence essentially all living organisms and affect many physiological processes from sleep and nutrition to immunity. This ability to respond to environmental daily rhythms has been conserved along evolution, and it is found among species from bacteria to mammals. The hematopoietic process of the crayfish *Pacifastacus leniusculus* is under circadian control and is tightly regulated by astakines, a new family of cytokines sharing a prokineticin (PROK) domain. The expression of AST1 and AST2 are light-dependent, and this suggests an evolutionarily conserved function for PROK domain proteins in mediating circadian rhythms. Vertebrate PROKs are transmitters of circadian rhythms of the suprachiasmatic nucleus (SCN) in the brain of mammals, but the mechanism by which they function is unknown. Here we demonstrate that high AST2 expression is induced by melatonin in the brain. We identify RACK1 as a binding protein of AST2 and further provide evidence that a complex between AST2 and RACK1 functions as a negative-feedback regulator of the circadian clock. By DNA mobility shift assay, we showed that the AST2-RACK1 complex will interfere with the binding between BMAL1 and CLK and inhibit the E-box binding activity of the complex BMAL1-CLK. Finally, we demonstrate by gene knockdown that AST2 is necessary for melatonin-induced inhibition of the complex formation between BMAL1 and CLK during the dark period. In summary, we provide evidence that melatonin regulates AST2 expression and thereby affects the core clock of the crustacean brain. This process may be very important in all animals that have AST2 molecules, i.e. spiders, ticks, crustaceans, scorpions, several insect groups such as Hymenoptera, Hemiptera, and Blattodea, but not Diptera and Coleoptera. Our findings further reveal an ancient evolutionary role for the prokineticin superfamily protein that links melatonin to direct regulation of the core clock gene feedback loops.

## Author Summary

Most living organisms are able to sense the time and in particular time of day by their internal clocks. So-called clock proteins control these internal clockworks. BMAL1 and CLK are two important clock proteins, which together form a complex that serves as a transcription factor and controls the production of diurnal proteins. These diurnal proteins, in turn, inhibit the formation of clock proteins so that the concentration of the different proteins in the cell oscillates back and forth throughout the day. External factors may affect the balance of clock proteins, and one such important factor is light. Melatonin is a darkness hormone produced in the brain of most animals during the night, and here we show that melatonin controls the formation of a protein named AST2 in crayfish. AST2 belongs to a group of proteins found in many arthropods, such as spiders, scorpions, crustaceans, and some insects, whose function has been unknown until now. Now we demonstrate that AST2 is induced by melatonin at night and then functions in the internal biological clock by preventing BMAL1 and CLK to form a complex. In this way, AST2 acts as a link between melatonin and the internal biological clock.

## Introduction

The physiology and behavior of most organisms are regulated according to daily environmental changes in a circadian manner. Circadian rhythms are often monitored by assaying behavioral and/or molecular fluctuations [1]. Clock genes and hormones are core regulators or pacemakers in circadian regulation, which reside in the suprachiasmatic nucleus (SCN) in mammals and the brain visual center in insects [2], [3]. In *Drosophila*, the proteins encoded by clock genes form two distinct heterodimers: Period (PER) and Timeless (TIM) form one heterodimer, and Clock (CLK) and Cycle (CYC) form the other [4]. In mammals, the homologues of the CLK and PER proteins have the same name, while the homologues of TIM and CYC are called cryptochrome (CRY) and brain and muscle aryl hydrocarbon receptor nuclear translocator (ARNT)-like 1 (BMAL1) respectively [5]. The PER-TIM heterodimer functions as an autoregulatory negative feedback loop that causes a decrease in transcriptional activation by CLK and CYC [6]. Conversely, the CLK-CYC heterodimer directly interacts with the upstream E-boxes (CACGTG) of the *PER* and *TIM* genes to activate their transcription [7]. These clock genes are detected in several neural and non-neural tissues, suggesting that these feedback loops are not restricted to neurons [8]. RACK1 was recently identified as an inhibitor of mammalian CLK-BMAL1 activity by recruiting PKCα during the negative feedback phase of the cycle [9].

As described above, the SCN serves as the “master clock” in the mammalian brain [10]. The SCN is reset on a circadian basis by light input from the retina during the day and by melatonin secretion from the pineal gland at night [11], [12]. Several animal studies have documented that melatonin is mainly synthesized and released during darkness, while the melatonin level is low in the presence of light [13]. This hormone is formed not only in the pineal gland but also in the photoreceptive structures of both vertebrates and invertebrates [14]. The melatonin synthesis pattern is known to reflect both daily rhythms and changes in photoperiod, demonstrating that melatonin has major roles in regulating both circadian and seasonal rhythms [15]. Several circadian rhythms, such as the rest/activity cycle, core body temperature, neuronal electrical activity and locomotor activity, are driven by melatonin [16], [17], [18], [19]. However, melatonin does not directly induce immediate changes in clock gene mRNA expression in the rat SCN, suggesting that the phase-shifting effect of melatonin on the SCN molecular loop implicates a post-translational rather than a transcriptional effect [15]. Little is known about the molecular mechanism by which melatonin drives the clock gene feedback loops in the SCN. In addition, the nocturnal increase in the circadian secretion of the cytokine IL-2 and its immunobiological activity are under melatonin control during the dark period [20]. There is a link between the rest/activity cycle and the immune system via melatonin-cytokine interactions [21].

Neuronal tissues that contain circadian clocks are present in the brain of the crayfish *Cherax destructor* and *Procambarus clarkii*, the latter of which is highly related to *Pacifastacus leniusculus*. These species have photoreceptor cells not only within their eyes, but also in extraretinal parts of the brain. In *Cherax* this area is located in the anterior median brain soma cluster 6 [22], and the axons from these cells terminate in an area within the protocerebral bridge [23]. It is clear that these brain photoreceptors are sufficient to maintain the circadian locomotor rhythm in these animals [23]. These areas have also recently been shown to be immunoreactive for proteins encoded by the clock genes CLK, PER and TIM [24]. Several studies imply a conserved role of melatonin as an important transducer of circadian information in invertebrates and vertebrates, and melatonin production has been demonstrated in the eyestalks of several crustacean species [25], [26]. The presence of MT2 melatonin receptors have not been conclusively shown in crayfish, but indirect evidences for such a receptor were presented by Mendoza-Vargas et al [27] since the application of the MT2 receptor selective agonist 8-M-PDOT or antagonist DH97 had a significant effect on how melatonin affected the retinal photoreceptors [27].

In mammals, the secretion of prokineticin 2 (PROK2) by the SCN is implicated in the regulation of the sleep/wake cycle and locomotor activity and is known to suppress the function of melatonin [28]. The transcription of PROK2 is activated by the CLK-BMAL1 heterodimer and light [29], [30].

Crayfish astakines are invertebrate homologues of the prokineticins (PROK), and there are two forms in the crayfish *P. leniusculus*: astakine 1 (AST1, AAX14635) and astakine 2 (AST2, EF568370) [31]. These astakines have been identified in several invertebrates, and similar to PROK2, the expression profiles of crayfish AST1 and AST2 follow a daily rhythm [32]. In contrast to AST1, the rhythmic expression of AST2 is at its maximum level in the dark phase [32]. Although the patterns of melatonin and AST2 release are circadian-regulated in crayfish [32], [33], nothing is known about their role in regulating rhythmic oscillations. In this study, we provide evidence that melatonin regulates the circadian rhythm and that this regulation is mediated by AST2 during the dark phase. Our results imply that AST2 acts as novel negative feedback regulator of CLK-BMAL1 activity.

## Results

### Melatonin induces the expression of AST2

In a recent report, we showed that AST2 mRNA is expressed in the hematopoietic tissue (HPT) of *P. leniusculus* at higher levels at night than during the day, the time when melatonin is also at a high level [32], [33]. Thus, we hypothesized that there may be a physiological link between these two molecules. We examined the expression of AST1 and AST2 in HPT cells incubated with melatonin *in vitro* (Figure 1A–1B) and in HPT, hemocytes and brain injected with melatonin *in vivo* (Figure 1C–1H). Melatonin incubation or injection clearly affected AST2 expression (Figure 1B, 1D, 1F and 1H), whereas AST1 expression was unaffected by this treatment (Figure 1A, 1C, 1E and 1G). These results were also confirmed at the level of translation using an ELISA assay (Figure 2A–2C), in which melatonin treatment resulted in higher levels of the AST2 protein. When cell lysates from the brain and HPT were analyzed by western blot at 9:00 and 20:00, respectively, the level of AST2 was clearly higher at night than during the day (Figure 2D).

**Figure 1:** AST2 expression is induced by melatonin treatment *in vitro* and *in vivo*. A) Relative expression of AST1 mRNA estimated by qPCR, after incubation with melatonin in cultured HPT cells *in vitro* at daytime. Black bars = melatonin (3 µM), white bars = control. B) Relative expression of AST2 mRNA estimated by qPCR, after incubation with melatonin in cultured HPT cells *in vitro* at daytime. Black bars = melatonin (3 µM), white bars = control. C) Relative expression of AST1 mRNA in hemocytes estimated by qPCR, after injection of melatonin in live crayfish. Black bars = melatonin (4.3 nmol/g), white bars = control. D) Relative expression of AST2 mRNA in hemocytes estimated by qPCR, after injection of melatonin in live crayfish at daytime. Black bars = melatonin (4.3 nmol/g), white bars = control. E) Relative expression of AST1 mRNA in HPT estimated by qPCR, after injection of melatonin in live crayfish at daytime. Black bars = melatonin (4.3 nmol/g), white bars = control. F) Relative expression of AST2 mRNA in HPT estimated by qPCR, after injection of melatonin in live crayfish at daytime. Black bars = melatonin (4.3 nmol/g), white bars = control. G) Relative expression of AST1 mRNA in the brain estimated by qPCR, after injection of melatonin in live crayfish at daytime. Black bars = melatonin (4.3 nmol/g), white bars = control. H) Relative expression of AST2 mRNA in the brain estimated by qPCR, after injection of melatonin in live crayfish at daytime. Black bars = melatonin (4.3 nmol/g), white bars = control. Expression of the 40S ribosomal protein was used as an internal control. Error bars indicate standard deviation (SD) from three replicates and the experiment has been repeated three times with similar results. The asterisks indicate significant differences (*P<0.05, **P<0.01); one-way ANOVA with Duncan's new multiple-range test and the Tukey test.

**Figure 2:** Melatonin induces higher AST2 protein levels *in vitro* and *in vivo*. A) Relative levels of AST1 or AST2 protein in cultured HPT cells *in vitro* as estimated by ELISA, after incubation with melatonin. Black bars = melatonin (3 µM), white bars = control. The level of β-actin was used as an internal control. B) Relative levels of AST1 in the HPT, brain and hemocytes in live crayfish as estimated by ELISA, after injection of melatonin. Black bars = melatonin (4.3 nmol/g), white bars = control. The level of β-actin was used as an internal control. C) Relative levels of AST2 in the HPT, brain and hemocytes in live crayfish as estimated by ELISA, after injection of melatonin. Black bars = melatonin (4.3 nmol/g), white bars = control. The level of β-actin was used as an internal control. The asterisks indicate significant differences (*P<0.05); one-way ANOVA with Duncan's new multiple-range test and the Tukey test. Results are representative of three independent experiments. Error bars indicate SD from three replicates and the experiment has been repeated three times with similar results. D) Western blot analysis of AST2 in the brain and HPT at 9:00 and 20:00, using an antibody against AST2. The expression level of actin was used as an internal control. Light and dark periods are indicated on the top of the blot.

### AST2 binds to *Pl*RACK1

In contrast to AST1, which is a secreted protein, AST2 is mainly an intracellular protein (Figure S1). To identify any protein that interacts with AST2 in HPT cells, recombinant AST2 (GST-AST2) was used as a bait to bind to proteins in HPT and hemocyte lysates by far overlay or pull-down assays (Figure 3A–3B). After excluding the background proteins found in the control, a protein with high similarity to *Penaeus monodon* RACK1 was identified as an AST2-binding protein by mass spectra analysis. The Mascot search resulted in significant hits where *P. monodon* RACK1 had the highest significant protein score 781 (Table S1). This protein was the significant hit detected in both the far overlay and the GST pull-down assay.

**Figure 3:** AST2 interacts with *Pl*RACK1. A) *Pl*RACK1 was identified as an AST2 binding protein using a far western assay with recombinant GST-AST2 or GST as a control. A HPT protein extract was subjected to SDS-PAGE, electroblotted to a PVDF membrane and overlayed with either GST (left) or GST-AST2 (right) alone and binding was detected using a GST antibody. B) The binding between recombinant AST2 with *Pl*RACK1 was confirmed by a GST pull-down assay using GST-AST2 as the binding protein and proteins in a HPT cell lysate as bait. GST was used as a control in both assays. C) GST pull-down of His-Trx-AST2 by GST-*Pl*RACK1. The bound proteins were analyzed by 12.5% SDS-PAGE. Bands corresponding to GST and GST-*Pl*RACK1 were detected with an anti-GST antibody (lanes 1–4). The eluted material was also examined for the presence of AST2 with an anti-His antibody (lanes 5–8). Lanes 9 and 10 contain purified His-Trx-AST2 and HisTrx, respectively.

By designing degenerate primers from the obtained amino acid sequences, a complete RACK1 cDNA was identified by RACE technique from *P. leniusculus* (*Pl*RACK1). The open reading frame of *Pl*RACK1 contains 957 bp (JQ686053), encoding 318 amino acids with a calculated molecular mass of 35.7 kDa (predicted MW using ProtParam program), and its deduced amino acid sequence was found to consist of seven conserved WD40 repeat binding sites (Figure S2). *Pl*RACK1 mRNA was highly expressed in different crayfish tissues (Figure S3). To confirm the interaction between *Pl*RACK1 and AST2, recombinant GST-*Pl*RACK1 was produced and purified with a predicted molecular mass of 62 kDa (Figure S5A). The GST-*Pl*RACK1 was used in an *in vitro* binding assay with a His-Trx-AST2 fusion protein (predicted mass of 33 kDa). The His-Trx and GST proteins were also expressed and purified to serve as control proteins (Figure S5B: the predicted mass of His-Trx and GST proteins are 20 and 26 kDa, respectively). As shown in Figure 3C, western blot analysis revealed that the His-Trx-AST2 protein was pulled down by GST- *Pl*RACK1, but not by GST alone. These data indicate that there is an interaction between *Pl*RACK1 and AST2.

### *Pl*BMAL1 forms a complex with *Pl*RACK1

The finding that *Pl*RACK1 is a binding partner of the melatonin-induced protein AST2 led us to examine whether *Pl*RACK1 associates with BMAL1 to thereby act as a regulator of circadian rhythm, as has recently been reported in mice [9]. BMAL1 cDNA was amplified from *P. leniusculus* (*Pl*BMAL1, JQ670886) with an open reading frame of 1,995 bp that encodes a 664 amino acid protein with a predicted molecular mass of 73.64 kDa. One close sequence to *Pl*BMAL1 was that of BMAL1 from *Drosophila melanogaster* (identity = 55%). Domain homology analysis using SMART revealed that the deduced amino acid sequence was highly conserved in its HLH (helix-loop-helix) DNA-binding domain and the protein dimerization PAS and PAC regions (Figure S4A). The expression of *Pl*BMAL1 was highest in hemocytes, followed by testis, nerve, intestine and brain (Figure S4B). An interaction between *Pl*BMAL1 and *Pl*RACK1 was demonstrated using a GST pull-down experiment with recombinant GST-*Pl*RACK1 (predicted mass of 62 kDa) and His-Trx-*Pl*BMAL1 (predicted mass of 94 kDa as shown in Figure S6A–S6B). This *in vitro* GST pull-down assay showed an apparent binding between these two recombinant proteins (Figure 4A). The far western blotting using *Pl*RACK1 without GST tag (predicted mass of 36 kDa) as a prey and GST- *Pl*BMAL1 (predicted mass of 100 kDa as shown in Figure S6C) as bait, also confirmed this interaction (Figure 4B). The results show that the GST-*Pl*BMAL1 was detected at the place where the *Pl*RACK1 was located, whereas the GST control protein could not be detected. Binding of *Pl*RACK1 to AST2 as well as to *Pl*BMAL1 was detected using far western after SDS-PAGE at reducing condition. The crystal structure of human RACK1, with high homology to *Pl*RACK1, is known as a sevenfold ß-propeller structure [34]. A comparison of the structure of human RACK1 with yeast RACK1 (that lacks most of the cysteines present in animal RACK1's) show a high similarity in the overall structure, indicating that the cysteines are of minor importance for the main structure characteristics of this group of proteins, which may explain retained binding properties in the far western assay.

**Figure 4:** *Pl*RACK1 can bind to *Pl*BMAL1. A) *In vitro* GST pull-down assay of His-Trx-*Pl*BMAL1 by GST-*Pl*RACK1. The elution fractions of the GST-*Pl*RACK1 pull-down assay were examined by western blot analysis using anti-GST and anti-His antibodies. Lanes 1 and 5: elution fraction of GST-*Pl*RACK1 pull-down of HisTrx-*Pl*BMAL1; Lanes 2 and 6: GST-*Pl*RACK1 pull-down of His-Trx; Lanes 3 and 7: GST pull-down of HisTrx-*Pl*BMAL1; Lanes 4 and 8; GST pull-down of His-Trx. B) The protein-protein interaction of *Pl*RACK1 and *Pl*BMAL1 was analyzed by far western blotting. C) Binding of AST2 and *Pl*BMAL1 to GST-*Pl*RACK1. GST-*Pl*RACK1 (0, 5, 50 or 500 ng) was bound to Glutathione Sepharose beads and incubated with 500 ng His-Trx-*Pl*BMAL1 and 500 ng His-Trx-AST2. Bound proteins were eluted and immunoblotted for *Pl*BMAL1 and AST2 using an anti-His antibody and for *Pl*RACK1 with an anti-GST antibody.

### Interaction of AST2 with *Pl*RACK1-*Pl*BMAL1 *in vitro*

To investigate if and how AST2 regulates an oscillatory mechanism, we examined whether AST2 interacts with the *Pl*BMAL1-*Pl*RACK1 complex. This interaction is mediated by AST2 binding to *Pl*RACK1, since we could show that AST2 is not able to bind to BMAL1 alone (Figure S7). The results from GST pull-down experiments showed that recombinant His-Trx-AST2 strongly associated with the recombinant GST-*Pl*RACK1/His-Trx-*Pl*BMAL1 complex, and the binding of His-Trx-*Pl*BMAL1 and His-Trx-AST2 was dependent on the concentration of GST-*Pl*RACK1 (Figure 4C). These results suggest that AST2 plays an essential role as a stabilizer of the *Pl*BMAL1-*Pl*RACK1 complex, thereby suppressing the CLK-BMAL1 interaction during the dark period.

### AST2 associates to form an AST2*-Pl*RACK1-*Pl*BMAL1 complex during the dark period *in vivo*

The amount of AST2 protein varies in a circadian manner and is highest during early night in the brain and HPT, while *Pl*BMAL1 and *Pl*RACK1 protein levels do not change significantly according to daily rhythms (Figure 5A–5B). Because our *in vitro* experiments indicated an interaction between AST2 and *Pl*RACK1 and between *Pl*RACK1 and *Pl*BMAL1, we confirmed these two interactions with *in vivo* experiments. To study the *in vivo* interactions between these three proteins during the light and dark periods, we performed immunoprecipitation experiments of brain and HPT extracts. A high-molecular-weight complex was present at night and disappeared during the day, as shown in Figure 5C and 5D. This complex was abundant in the brain; it was also found at very low levels in a few HPT samples (Figure 5C). Reducing SDS-PAGE revealed that AST2, *Pl*BMAL1 and *Pl*RACK1 were components of this approximately 200 kDa complex (Figure 5C) (the native mass of these three proteins are 14, 74 and 36 kDa, respectively). During the light period, this high molecular weight complex could not be detected; instead, a smaller complex of AST2-*Pl*RACK1 was identified (Figure 5D).

**Figure 5:** *Pl*RACK1, *Pl*BMAL1, and AST2 form an approximately 200-kDa protein complex during the dark period. A) Relative amounts of AST2, *Pl*RACK1 and *Pl*BMAL1 proteins in brain extracts as determined by ELISA at 3 h after light turned off or on. B) Relative amounts of AST2, *Pl*RACK1 and *Pl*BMAL1 proteins in HPT extracts as determined by ELISA at 3 h after light turned off or on. The asterisks indicate significant differences (*P<0.05); one-way ANOVA with Duncan's new multiple-range test and the Tukey test. Results are representative of three independent experiments. Error bars indicate SD from three replicates and the experiment has been repeated three times with similar results. C) Immunoprecipitation (IP) of brain extract using antibodies against RACK1, BMAL1 and AST2 revealed that a *Pl*RACK1-AST2 complex was present in the brain (B) during the day. D) Immunoprecipitation (IP) of brain extract using antibodies against RACK1, BMAL1 and AST2 revealed the presence of a high-molecular-weight complex (approximately 200 kDa) composed of all three proteins in the brain (B) at night. C–D) The immunoprecipitated complex was analyzed by western blotting (WB) using another antibody. “B” and “HPT” represent brain and hematopoietic tissue, respectively. The antibodies used for immunoprecipitation (IP) and detection (WB) is indicated at the top and bottom of the blots, respectively, and +DTT and −DTT represent reducing and non-reducing conditions, respectively. Molecular masses are indicated at the left.

### The CLK protein is detected as a component of the 400-kDa complex

To determine whether CLK (JQ670885) forms a complex with BMAL1, crayfish brain lysates were prepared, immunoprecipitated with antibodies against BMAL1 and probed for CLK. The CLK protein with a molecular mass of 95 kDa clearly coimmunoprecipitated with endogenous *Pl*BMAL1 (Figure 6A), indicating that CLK is one protein component of this large approximately 400 kDa complex. Confirmation of complex formation was accomplished by switching the antibodies used for immunoprecipitation and for western blot detection, respectively (Figure 6A). We then monitored the CLK protein levels in the brain during the day and night by western blotting. As shown in Figure 6B, the CLK protein level oscillated in a circadian rhythm, and its expression peaked in the light period (Figure 6F). Furthermore, the approximately 400 kDa CLK-*Pl*BMAL1 complex was barely detectable at night and reached maximal levels in the morning (Figure 6B and 6C). More interestingly, the lowest level of the CLK-*Pl*BMAL1 complex in brain lysates coincided with the time at which the AST2*-Pl*RACK1-*Pl*BMAL1 complex was at its highest level (Figure 6B and 6D). Thus, these data indicate that AST2 is an important regulator of circadian rhythm by interfering with formation of the CLK-*Pl*BMAL1 complex.

**Figure 6:** A 400-kDa CLK-*Pl*BMAL1 complex is present in the light in the crayfish brain. A) Immunoprecipitation (IP) of endogenous CLOCK (CLK) and *Pl*BMAL1 in the brain (B) and HPT. Total proteins were extracted from the brain and HPT and were immunoprecipitated (IP) with the antibodies (Ab) indicated on the top of the blots, followed by western blot (WB) detection with antibodies against CLK or BMAL1 as shown at the bottoms of the blots. Reducing and non-reducing conditions of the samples are indicated by +DTT or −DTT, respectively. B) The levels of the CLK-*Pl*BMAL1 and AST2-*Pl*RACK1-*Pl*BMAL1 protein complexes were analyzed by SDS-PAGE under non-reducing conditions (sample without DTT) followed by western blotting using an antibody against BMAL1. The AST2-*Pl*RACK1 heterodimer and CLK were detected by western blotting using antibodies against AST2 and CLK, respectively. Time points were taken at 03:00, 06:00, 12:00, 18:00, and 21:00 (n = 4). An actin protein was used as an internal control. The horizontal band at the top of the histogram indicates the light condition (white = light, black = dark). C) Relative amounts of CLK-*Pl*BMAL1 protein complex in brain extracts at different time points (n = 3) as determined by western blotting. D) Relative amounts of AST2-*Pl*RACK1-*Pl*BMAL1 protein complex in brain extracts at different time points (n = 3) as determined by western blotting. E) Relative amounts of AST2-*Pl*RACK1 protein complex in brain extracts at different time points (n = 3) as determined by western blotting. F) Relative amounts of CLK protein in brain extracts at different time points (n = 3) as determined by western blotting. Average protein level in Graphs C–F was quantitated using Quantity One. The asterisks indicate significant differences (*P<0.05, **P<0.01); one-way ANOVA with Duncan's new multiple-range test and the Tukey test. Results are representative of three independent experiments. Error bars indicate SD from three replicates and the experiment has been repeated three times with similar results. G) Melatonin injection inhibited the formation of the CLK-*Pl*BMAL1 complex; this inhibition is mediated by the AST2-*Pl*RACK1-*Pl*BMAL1 complex. The levels of the CLK-*Pl*BMAL1 and AST2-*Pl*RACK1-*Pl*BMAL1 protein complexes were analyzed by SDS-PAGE under non-reducing conditions (sample without DTT) followed by western blotting using an antibody against BMAL1. The level of β-actin was used as an internal control. H) Relative levels of CLK-*Pl*BMAL1 and AST2-*Pl*RACK1-*Pl*BMAL1 complexes *in vivo*, in the brain of crayfish after injection of melatonin and then brain extracts were analyzed by western blotting using an antibody against BMAL1. Grey bars = melatonin (4.3 nmol/g), white bars = control injection (PBS). I) Relative levels of CLK-*Pl*BMAL1 and AST2-*Pl*RACK1-*Pl*BMAL1 complexes *in vivo*, in the HPT of crayfish after injection of melatonin and then HPT extracts were analyzed by western blotting using an antibody against BMAL1. Grey bars = melatonin (4.3 nmol/g), white bars = control injection (PBS). The level of β-actin was used as an internal control. Asterisks indicate significant differences (*P<0.05, **P<0.01). Quantity One analysis was used to quantify the intensity of protein bands. Graphs (H and I) represent the quantification of each complex formation, using Quantity one. Results are representative of three independent experiments. Statistical significance: *P<0.05, **P<0.01 using Student's paired t-test (error bars indicate SD from nine replicates).

### The effect of melatonin injection during the light period

Because we detected a clear stimulatory effect of melatonin on the expression of AST2 (Figure 2C), we decided to further confirm this putative role of AST2 by determining the presence, *in vivo*, of the approximately 400 kDa CLK-*Pl*BMAL1 and approximately 200 kDa AST2*-Pl*RACK1-*Pl*BMAL1 complexes, respectively, after melatonin injection during the light period. Six hours after melatonin injection, the approximately 200 kDa complex was detected in the crayfish brains, but not in the HPT (Figure 6G–6I). Conversely, the amount of the approximately 400 kDa complex containing CLK-*Pl*BMAL1 was reduced post-melatonin injection (Figure 6G and 6H). These results indicate that either secretion of natural melatonin at night or melatonin treatment causes an increase in the AST2 protein level and thereby increases the amount of the approximately 200 kDa complex.

### AST2 is required for delayed CLK-BMAL1 formation

To further test whether AST2 is crucial for the interference of CLK-BMAL1 heterodimer formation, AST2 mRNA expression was partially knocked down by RNAi, to ca 50% of the control. As shown in Figure 7A and 7B, AST2 expression could be partly decreased in the brain by injection of dsRNA. A reduction of the approximately 200 kDa complex occurred during the night as a result of this AST2 deficiency when compared to injection of the dsGFP control (Figure 7C and 7E). In contrast to the control group, the formation of the ≈400 kDa complex in AST2-silenced animals occurred at 21:00, as shown in Figure 7C and 7D. Thus, this experiment further confirms that AST2 is required to interfere with the formation of the CLK-*Pl*BMAL1 heterodimer, and that high AST2 levels at night cause lower amounts of CLK-*Pl*BMAL1 heterodimer formation during the dark period (Figure 7C–7G).

**Figure 7:** AST2 is required to regulate the CLK-*Pl*BMAL1 heterodimer formation. A) The relative expression levels of AST2 in the brain at 03:00, 06:00, 12:00, and 21:00 (n = 9) after partial knock down of AST2 (grey) in the brain by dsRNA injection and detection by qPCR; dsGFP injection was used as a control (white). B) The relative expression levels of AST2 in hemocytes at 03:00, 06:00, 12:00, and 21:00 (n = 9) after partial knock down of AST2 (grey) by dsRNA injection and detection by qPCR; dsGFP injection was used as a control (white). Graph A and B represent AST2 mRNA levels, using qPCR. Results are representative of three independent experiments. Error bars indicate SD of nine replicates. The asterisks indicate significant differences (*P<0.05, **P<0.01); Student's paired t-test. C) The effect of dsAST2 on complex formation in the brain *in vivo* was examined by western blotting of brain extracts and detection as follows: for the CLK-*Pl*BMAL1 complex an anti-BMAL1 antibody, for the AST2- *Pl*RACK1-*Pl*BMAL1 complex an anti-BMAL1 antibody, and for the AST2-*Pl*RACK1 an anti- AST2 antibody was used. The horizontal band at the top of the histogram indicates the light condition (white = light, black = dark). D) Relative amounts of CLK-*Pl*BMAL1 protein complex in the brain *in vivo* was determined at different time points (n = 9) by western blotting of brain extracts, using an antibody against BMAL1. Grey bars = dsAST2, white bars = dsGFP. E) Relative amounts of AST2-*Pl*RACK1-*Pl*BMAL1 protein complex in the brain *in vivo* was determined at different time points (n = 9) by western blotting of brain extracts, using an antibody against BMAL1. Grey bars = dsAST2, white bars = dsGFP. F) Relative amounts of AST2-*Pl*RACK1 protein complex in the brain *in vivo* was determined at different time points (n = 9) by western blotting of brain extracts, using an antibody against RACK1. Grey bars = dsAST2, white bars = dsGFP. G) Relative amounts of AST2 protein in the brain *in vivo* was determined at different time points (n = 3) as determined by western blotting of brain extracts, using an antibody against AST2. Grey bars = dsAST2, white bars = dsGFP. Quantity One analysis was used to quantify the intensity of protein bands from three independent experiments and results are presented in graphs D to G. Statistical significance: *P<0.05, **P<0.01 using Student's paired t-test (error bars indicate SD from nine replicates).

### AST2 gene knockdown induces CLK/BMAL1 E-box binding in the dark

Since knockdown of AST2 resulted in more CLK-*Pl*BMAL1 complex formation during the dark period, we decided to test whether AST2 also had an effect on CLK-*Pl*BMAL1 E-box binding. We assayed the CLK-*Pl*BMAL1 E-box binding by a DNA-protein binding assay. As expected, we could demonstrate CLK-*Pl*BMAL1 specific E-box binding during the night in AST2 silenced animals, whereas the control group (dsGFP) did not show any E-box binding in the dark (Figure 8A–8B). A super shift of this E-box binding was induced after incubation with anti-CLK antibodies (Figure 8A), and controls using mutated or unlabelled E-box oligonucleotides did not show any binding (Figure 8B and Figure S8A–S8B). In contrast, melatonin injection during the day (which leads to enhanced levels of AST2, Figure 2A) reduced the DNA binding activity of CLK-*Pl*BMAL1 compared to other groups (Figure S8B). The complex formation of CLK-*Pl*BMAL1 or AST2*-Pl*RACK1-*Pl*BMAL1 was followed by western blotting after knockdown of AST2 expression by dsRNA or increasing AST2 by addition of melatonin (Figure 8C–8E). These results reveal that AST2 is an important regulator of the E-box binding activity of the CLK-*Pl*BMAL1 complex.

**Figure 8:** AST2 knockdown enhanced the DNA binding activity of CLK/*Pl*BMAL1. A) Crayfish received dsGFP or dsAST2 treatments, then crude brain lysates were harvested during day and night, and were used to study E-box binding with fluorophore labeled oligonucleotides in an EMSA assay. As a control the brain lysates were incubated with an antibody against CLK, to show a supershift. The E-box binding activity of CLK-*Pl*BMAL1 is indicated on the right side of the gel. B) The effect of AST2 knock down on CLK-*Pl*BMAL1 E-box binding was analyzed by EMSA. A mutant E-box was used as control. C) Western blot showing the effect of AST2 knock down or melatonin treatment on the protein levels of CLK/*Pl*BMAL1, AST2-*Pl*RACK1-*Pl*BMAL1 complexes (upper panel), and AST2 level (middle panel). Actin was used as an internal control (lower panel). The horizontal band on top of this histogram indicates day (white) or night (black). D) Relative amounts of CLK-*Pl*BMAL1 and AST2*-Pl*RACK1-*Pl*BMAL1 protein complexes in brain extracts isolated during the day (n = 9) as determined by western blotting, using an antibody against BMAL1. The AST2 protein was also detected by western blotting, using an antibody against AST2. White bars = dsAST2, black bars = melatonin, grey bars = dsGFP. E) Relative amounts of CLK-*Pl*BMAL1 and AST2*-Pl*RACK1-*Pl*BMAL1 protein complexes in brain extracts isolated during the night (n = 9) as determined by western blotting, using an antibody against BMAL1. The AST2 protein was also detected by western blotting, using an antibody against AST2. White bars = dsAST2, and grey bars = dsGFP. In three independent experiments, proteins were visualized by western blotting and quantitated using the Quantity One software. These results are shown in graph D and E. Error bars indicate SD from nine replicates. The asterisks indicate significant differences (*P<0.05, **P<0.01); one-way ANOVA with Duncan's new multiple-range test and the Tukey test.

## Discussion

Various proteins are regulated by the circadian rhythm, and there are a growing number of examples of circadian regulation of stem cell activities, such as the proliferation and recruitment of hematopoietic progenitor cells [33], [35]. We have recently shown that the hematopoietic cytokine AST1 is regulated by light and that this regulation has an impact on hemocyte synthesis [26]. AST1 contains a prokineticin domain (pfam06607) and shares similarities with vertebrate PROK2, which is regulated by light at the transcriptional level by core clock genes [22]. Apart from functioning in circadian clocks, vertebrate PROKs have documented roles in the regulation of intestinal muscle contractility, neurogenesis, pain perception, food uptake, and appetite regulation [36], [37]. In similarity with invertebrate astakines the vertebrate PROKs also play roles in hematopoiesis and proinflammatory immune responses. Therefore, the structural and functional similarities between astakines and the vertebrate PROKs point to an ancient similar role for these proteins [38].

The oscillation in PROK2 transcription in mice occurs in the SCN, and it acts as an output molecule, signaling the rhythm to other cells and tissues and thereby changing circadian behavior [39]. Signal transduction from vertebrate PROK's are mediated by two closely related G-protein coupled receptors, and the AVIT motif has been shown to be crucial to this receptor binding and the activity of the PROK's [40]. An analysis of the gene structure for human PROK2 reveals that exon 2–4 share similarities to crayfish AST2, while the first exon encodes the signal peptide and the AVIT motif [41], [42]. Thus, all invertebrate astakines found so far, differ from the vertebrates PROKs in their N-terminal and lack of the AVIT-motif [25] a fact that indicates different receptor binding properties for this invertebrate group of PROK domain containing proteins. Similar to PROK2, AST1 is a secreted molecule with circadian expression, and these data indicate a conserved role for this domain throughout evolution, from arthropods to humans [25], [26]. In this study, we report a more direct role for another crayfish prokineticin, namely AST2, as an intracellular regulator of the heterodimeric transcription factors CLK and *Pl*BMAL1. The expression of AST2 does not exhibit a light-dependent pattern that is similar to that of AST1 or PROK2 in mice; instead, we detected high levels of AST2 expression in the HPT and brain during the dark period when melatonin levels are high. We also showed that melatonin administration clearly increased the expression of AST2 at both the mRNA and protein levels.

It is well established that the neurohormone melatonin has an important function in the SCN in regulating the feedback loop of the core clock genes and also functions as an output signal that has an effect on peripheral cells [43]. Melatonin is mainly produced within the eyestalks of crayfish, and its production is elevated during the dark period [27]. Melatonin is known to influence numerous physiological processes in crayfish [18], [33], [44], although the molecular mechanism by which melatonin exerts its effect has not been fully clarified. However, AST2 is an intracellular protein that is present in several crustaceans and insect species [25]. Here, for the first time, we identify a direct role for AST2 in the regulation of the circadian clock and show that the protein acts as a link between melatonin and the heterodimeric transcriptional activator CLK-*Pl*BMAL1. Intracellular *Pl*RACK1 was identified as an AST2-binding protein, and in the brain, the binding of *Pl*BMAL1 to this complex mediated a decrease in the formation of the CLK-*Pl*BMAL1 heterodimer. This process may be very important in all animals that have AST2 molecules i.e., spiders, ticks, crustaceans, scorpions, several insect groups such as Hymenoptera, Hemiptera, Blattodea but not Diptera and Coleoptera. If any vertebrate PROK is performing the same function still remains to be demonstrated.

Recently, RACK1 and protein kinase Cα (PKCα) were shown to interact with BMAL1 in a circadian manner, resulting in suppressed CLK-BMAL1 activity [9]. This result is consistent with our observation of the *Pl*RACK1-*Pl*BMAL1 interaction in the crayfish brain. At night, we detected an approximately 200 kDa complex in the crayfish brain and found that the components of this complex consisted of AST2, *Pl*RACK1 and *Pl*BMAL1. Conversely, this complex disappeared during the light period due to lower levels of AST2 during the day. Thus, our results show that AST2 acts as a regulator of the CLK-*Pl*BMAL1 complex by binding to *Pl*RACK1-*Pl*BMAL1 in an oscillatory manner that is induced by changes in the level of melatonin.

Interestingly, enhancement of the approximately 400 kDa complex consisting of *Pl*BMAL1 and CLK was detected when the level of the approximately 200 kDa complex was decreased either during the light period or by knockdown of AST2 expression. A similar high-molecular-weight complex of *Pl*BMAL1 and CLK (approximately 400 kDa) was also recently detected in mice [9]. The formation of the approximately 400 kDa crayfish complex is dependent on the expression of CLK. The expression of mammalian CLK is not rhythmic [45], [46], while zebrafish CLK shows robust rhythmic expression, as was the case for crayfish CLK in our study [47], [48], [49]. As with zebrafish and *Drosophila*, the CLK of crayfish is directly regulated by light [50], [51]. Unlike those in mammals, the protein products of *PER* and *TIM* (or *CRY* in mammals) in *Drosophila* act to inhibit the transcriptional activity of the CLK-CYC complex (CLK-BMAL1) by interacting with CLK or a CLK-containing complex during the night but not during most of the day [52]. In our experiments, the AST2-*Pl*RACK1-*Pl*BMAL1 complex (approximately 200 kDa) competes for binding to *Pl*BMAL1 to interfere with the formation of the CLK-*Pl*BMAL1 heterodimer during the dark period. Further it is clear from our DNA mobility shift assay that AST2 can inhibit the transcriptional activation activity of CLK-*Pl*BMAL1. This 200 kDa AST2-containing complex directly interacts with different proteins and is clearly induced by melatonin. Therefore, our findings reveal an ancient evolutionary role for a prokineticin superfamily protein that links melatonin to direct regulation of the core clock gene feedback loops, as indicated in the model (Figure 9).

**Figure 9:** Molecular model of the circadian regulation by CLK, *Pl*BMAL1, *Pl*RACK1, and AST2. The protein level of CLK is enhanced during the light period, and a CLK-*Pl*BMAL1 complex is formed that acts as a transcriptional activator. During the dark period melatonin secretion causes an upregulation of AST2 and this high AST2 level results in the formation of a complex between *Pl*BMAL1 and *Pl*RACK1. Then AST2 binds to PlRACK 1 in the PlBMAL-PlRACK1 complex and forms the AST2-*Pl*RACK1-*Pl*BMAL1 complex and this interferes with the formation and activity of the CLK-*Pl*BMAL1 heterodimer.

## Materials and Methods

### Crayfish

Healthy intermolt freshwater crayfish (*P. leniusculus*) were obtained from Lake Hjälmaren, Sweden and were maintained in aerated tap water at 10°C.

### Cloning and sequence analysis of full-length *P. leniusculus* RACK1 (*Pl*RACK1) and *Pl*BMAL1 cDNAs

Total RNA was isolated from crayfish brains using TRIzol LS (Invitrogen) followed by RNase-free DNase I (Ambion) treatment. cDNA synthesis was accomplished with an oligo (dT) primer and ThermoScript RT-PCR (Invitrogen) according to the manufacturer's protocol. A partial sequence of *Pl*RACK1 was amplified using primers that were designed based on the shrimp (*P. monodon*) *Pm*RACK1 sequence (GenBank accession no. EF569136), whereas *Pl*BMAL1 primers were based on the cDNA sequences from several organisms (listed in Table S2). To obtain the full-length cDNAs of the *Pl*RACK1 and *Pl*BMAL1 genes, 5′ and 3′ rapid amplification of cDNA ends (RACE) technology was performed using the SMARTer RACE cDNA Amplification Kit (Clontech) according to the manufacturer's instructions. The complete *Pl*RACK1 cDNA sequence was amplified using gene-specific primers for *Pl*RACK1 (Table S2) and the SMART Universal Primer A. The PCR products were then cloned into the TOPO TA cloning vector and sequenced. The deduced amino acid sequence of the *Pl*RACK1 gene was searched against the GenBank database with the BLAST program (http://www.ncbi.nlm.nih.gov/BLAST/). Sequence alignment of *Pl*RACK1 was generated by ClustalW, and the protein domains were analyzed with the SMART program (http://smart.embl-heidelberg.de/).

### Tissue distribution analysis

Total RNAs were isolated from different crayfish tissues using TRIzol reagent (Invitrogen) followed by RNase-free DNase I (Ambion) treatment. For reverse transcription, 1 µg of total RNA was reverse transcribed to produce cDNA using ThermoScrip RT-PCR (Invitrogen). To amplify and visualize the cDNAs of *Pl*RACK1 and *Pl*BMAL1, two sets of primers were used: the forward and reverse primers listed in Table S2. The PCR cycles were as follows: 1 cycle (95°C for 2 min); 28 cycles (95°C, 30 s; 55°C, 30 s; 72°C, 40 s) followed by an extension step (72°C for 5 min). The transcription of the 40S ribosomal protein was used as an internal control. All PCR products were analyzed on 1% GelRed-stained agarose gels.

### Crayfish HPT cell culture and maintenance

The hematopoietic tissue was dissected, washed with CPBS (crayfish phosphate buffered saline (pH 6.8), 10 mM Na_2_HPO_4_, 10 mM KH_2_PO_4_, 150 mM NaCl, 10 µM CaCl_2_, and 10 µM MnCl_2_,) and incubated in 600 µl of 0.1% collagenase (types I and IV) (Sigma) in CPBS at room temperature for 45 min to separate the HPT cells. The separated cells were washed twice with CPBS by centrifugation at 800×g for 5 min at room temperature. The cell pellet was re-suspended in modified L-15 medium, and cells were then seeded at a density of 2.5×10^6^ cells/150 µl in 96-well plates. The HPT cells were supplemented with partially purified plasma as a source of AST1 after 1 h of attachment at room temperature. The culture plates were incubated at 16°C, and 1/3 of the medium was changed at 48 h intervals.

### Melatonin treatment

For the *in vivo* experiments, 100 µl of a melatonin solution (Sigma) was dissolved in ethanol and diluted in crayfish saline (to a final ethanol concentration of 1%). This solution was injected into the base of a walking leg such that the amount of injected melatonin was 4.3 nmol/g fresh weight. Control crayfish received 100 µl of saline with 1% ethanol. The hemolymph, brain, and HPT of these crayfish were collected at 0, 1, 2, 3, and 6 h post-injection for the extraction of total RNA, whereas samples for total protein extraction were dissected at 3 h post-injection. All injections were performed during the day.

For the *in vitro* experiments, HPT cell cultures were prepared and incubated at 16°C for 12 h. The medium was then replaced with 150 µl of L-15 medium containing 5 µl of the melatonin solution at final concentration of 0.43 nmol/well (3 µM) (the control group was supplemented with 5 µl of saline with 1% ethanol) and 5 µl of crude AST1, followed by incubation for 0, 0.25, 1, 3, 6, and 12 h at 20°C. Thereafter, the cells were harvested at each time point for extraction of total RNA and protein. The transcription and translation levels of AST1 and AST2 *in vitro* and *in vivo* were detected by quantitative RT-PCR and ELISA, respectively.

### Sampling times

The light in the aquarium room was turned on and off at 4:00 and 20:00, respectively. Brains were dissected at 06:00, 12:00, 16:00, 21:00, and 03:00 from three crayfish at each sampling time, which were kept in normal light/dark conditions. The experiments were repeated at least twice. Complex formation and CLK expression were determined by western blotting using antibodies against BMAL1 and CLK, respectively. An anti-actin antibody (Santa Cruz Biotechnology) was used as an internal control.

### Generation of dsRNA

A T7 promoter sequence was incorporated into gene-specific primers for AST2 and GFP (italic letters) at their 5′ ends (AST2 RNAi-F, 5′- *TAA TAC GAC TCA CTA TAG GG*T CCA CGC CTC TGA GTC TTT T-3′; AST2 RNAi-R, 5′- *TAA TAC GAC TCA CTA TAG GG*A TGC CCA GAG TGT TGT CCT C-3′ and GFP 63+, 5′- *TAA TAC GAC TCA CTA TAG GG*C GAC GTA AAC GGC CAC AAG T-3′; GFP 719-, 5′- *TAA TAC GAC TCA CTA TAG GG*T TCT TGT ACA GCT CGT CCA TG-3′). These primers were used to amplify PCR products as templates for dsRNA synthesis. A GFP transcript was amplified with the pd2EGFP-1 vector (Clontech) as a template and was used as a control. The amplified products were then purified using a GenElute Gel extraction kit (Sigma) followed by *in vitro* transcription using a MegaScript kit (Ambion), and the dsRNA was purified with TRIzol LS (Invitrogen).

### dsRNA *in vivo*

Small intermolt crayfish (15±2 g of fresh weight) were divided into two groups with three crayfish in each group (n = 3). The first and second groups were injected with 300 µg of GFP control dsRNA and 300 µg of dsAST2, respectively, at the base of the fourth walking leg. Twenty-four hours after the first dsRNA injection, four drops of crayfish hemolymph were bled for total RNA isolation to test the efficiency of the RNAi. Then, dsRNA was injected a second time into both groups as described above. Twenty-four hours after the second dsRNA injection, the brains were dissected at 06:00, 12:00, 21:00, and 03:00 to determine complex formation by western blotting.

### Plasmid constructs

*Pl*RACK1 was amplified using the synthesized forward primer RACK1_F1 and reverse primer RACK1_R1 (Table S2) by PCR. The conditions for the PCR reactions were essentially identical to those described in the manufacturer's protocol for the vector. All constructs were sequence-verified. The PCR product was cloned into the pGEX-4T-1 bacterial expression vector at the *Bam*HI and *Sal*I cleavage sites.

*Pl*BMAL1 was amplified from crayfish testis cDNA by PCR using 1 unit of Paq5000 DNA polymerase (Stratagene) and a pair of specific primers listed in Table S2. *Eco*RI and *Xho*I sites were engineered into the primers to facilitate subsequent cloning. *Pl*BMAL1 was further subcloned into the pGEX-4T-1 and pET-32a vectors. The recombinant plasmids containing the *Pl*RACK1 and *Pl*BMAL1 genes were confirmed by DNA sequencing.

### Bacterial protein expression and purification

The full-length cDNA encoding *Pl*RACK1was cloned into the pGEX-4T-1 bacterial expression vector to express a glutathione S-transferase (GST)-fused *Pl*RACK1 protein in the *Escherichia coli* strain BL21(DE3). Protein expression was induced by adding IPTG to a final concentration of 1 mM at 25°C for 6 h. The cells were harvested by centrifugation followed by suspension in lysis buffer (50 mM NaH_2_PO_4_ (pH 8.0), 300 mM NaCl and 2% Triton X-100) and lysis by sonication. Inclusion body pellets were solubilized in denaturing buffer (50 mM Tris (pH 8.0), 8 M guanidine (GdnHCl) and 10 mM DTT) followed by centrifugation (13,000 rpm for 15 min). The protein was refolded in refolding buffer (55 mM Tris-HCl, 0.44 M L-arginine, 21 mM NaCl, 0.88 mM KCl and 10 mM DTT). The refolded GST-*Pl*RACK1protein was dialyzed in phosphate-buffered saline (PBS, pH 7.4) and applied to Glutathione Sepharose 4B resin (Amersham Biosciences, Inc.) for 30 min at room temperature. The beads were washed with ice-cold PBS followed by incubation in reducing buffer (50 mM Tris-HCl and 20 mM reduced glutathione, pH 8.0) for 30 min at room temperature. After centrifugation at 1,000×*g* for 5 min, the supernatant was collected and analyzed by 12.5% SDS-PAGE. The protein concentration was measured, and the proteins were stored at −80°C. The full-length sequence of *Pl*BMAL1 was ligated into *Eco*RI/*Xho*I-linearized pGEX-4T-1 and pET-32a vectors to create a plasmid that expresses GST- and His-Trx fusion proteins, respectively. The recombinant GST-*Pl*BMAL1 protein was expressed and purified in a similar manner as the GST-*Pl*RACK1 protein. The His-Trx-*Pl*BMAL1 recombinant protein was purified using a Ni-NTA column. His-Trx-AST2 was expressed and purified as described in earlier publications [25]. Briefly, His-Trx tagged AST2 was expressed in *E. coli* BL21 (DE3) and induced by the addition of 0.02 mM IPTG. The cells were resuspended in lysis buffer (50 mM NaH_2_PO_4_, pH 8.0, 300 mM NaCl and 2% Triton X-100) and purified using HisPur Cobalt Resin (Thermo Scientific). The protein products of the His-Trx tag expression vector pET-32a and the expression vector pGEX-4T-1, which are used for the incorporation of N-terminal thioredoxin and GST tags, respectively, were expressed in *E. coli* BL21(DE3) cells. The thioredoxin and GST proteins were purified with HisPur Cobalt or Glutathione Sepharose resins, respectively, as control proteins. All samples were analyzed by 12% SDS-PAGE.

### *In vitro* GST pull-down assay

To identify putative AST2-binding proteins, total protein was extracted from crayfish brains in buffer containing 50 mM Tris-HCl (pH 7.2), 100 mM NaCl, 10% glycerol, 1 mM PMSF, 10 µM MG132 and Complete Mini Protease Inhibitor tablets according to the manufacturer's instructions (Roche Diagnostics). Cell debris was removed by centrifugation at 10,000×g for 10 min. Recombinant GST–AST2 was expressed in *E. coli* and purified using glutathione Sepharose 4B resin according to standard protocols. GST–AST2 or GST (3–4 µg) was incubated with 800 µg of crude brain total protein extract at 4°C for 1 h unless otherwise specified. Glutathione beads were recovered by brief centrifugation and washed three times with 1 ml of washing buffer (50 mM Tris-HCl (pH 7.2), 100 mM NaCl, 10% glycerol and 0.1% Tween 20). GST was used as a control protein in this experiment. Pull-down mixtures were separated by SDS–PAGE, and after excluding the background proteins found in the control, the remaining band of about 30 kDa was sequenced by mass spectrometry after trypsin cleavage. Identification of the protein was based on raw MS/MS data, and ions search using the Mascot program (http://www.matrixscience.com).

The interaction between GST-*Pl*RACK1and HisTrx-AST2 was examined by incubating purified GST-*Pl*RACK1or the GST control with Glutathione Sepharose 4B resin (50 µl a 50% bed slurry) at room temperature for 1 h. The beads were washed three times with PBS, purified HisTrx-AST2 or the His-Trx control (5 µg) was added, and incubated for another 2 h at room temperature in PBS buffer. After washing with PBS, the precipitated proteins were eluted with SDS-sample buffer.

To determine the formation of a *Pl*RACK1-*Pl*BMAL1 complex, 5 µg purified His-Trx-*Pl*BMAL1 protein was incubated with 5 µg purified GST-*Pl*RACK1 protein bound to Glutathione Sepharose 4B beads. The beads were then washed five times, and the remaining proteins were eluted with SDS-sample buffer.

To explore whether AST2 can bind to *Pl*RACK1 together with *Pl*BMAL1, purified His-Trx-*Pl*BMAL1 (500 ng) and His-Trx-AST2 (500 ng) were incubated with Glutathione Sepharose 4B-bound GST-*Pl*RACK1 (0, 5, 50, 500 ng) in PBS buffer at 25°C for 2 h. The protein-bead complexes were washed, and the bound proteins were eluted with SDS-sample buffer. All protein samples were resolved by SDS-PAGE and were analyzed by western blot.

### Blot overlay assays

In addition to an *in vitro* GST pull-down assay, a far western overlay assay was used to identify any putative AST2 binding protein. The protein was extracted from crayfish HPT and then subjected to 12% SDS-PAGE, transferred to PDVF membranes, and blocked with 10% skim milk in TBST buffer (10 mM Tris-HCl (pH 7.5), 150 mM NaCl and 0.05% Tween 20) at room temperature. After three washes with TBST, the membranes were incubated with 25 mM GST-AST2 or GST alone in 10 ml TBST buffer at room temperature. The blots were washed twice and incubated for 1 h with 1∶2,000 dilution of anti GST antibody and then washed twice, incubated for 1 h with 1∶1,000 dilution of anti mouse antibody for 1 h, and washed three times before detection with an ECL western blotting reagent kit. The control reaction was incubated with GST instead of GST-AST2.

Purified GST-*Pl*RACK1 protein was cleaved by incubation with thrombin (GE Healthcare, 1 µl thrombin per 100 µg recombinant protein) at 22°C overnight to remove the GST fusion tag. Free *Pl*RACK1was eluted with PBS from the Glutathione Sepharose 4B beads. *Pl*RACK1 was run on 12.5% SDS-PAGE, transferred to PDVF membranes and incubated at 4°C overnight with purified GST-*Pl*BMAL1 or GST alone (7 µg) in 10 ml TBST buffer. The blot was washed three times (10 min each) in TBST containing 0.05% Tween 20. Protein interactions were detected by western blotting using an anti-GST antibody. Blot overlay assays were also used to confirm the binding of AST2. Preparation of total crayfish brain homogenates and gel overlays with recombinant GST-AST2 (far western blots) were performed as described above.

### Protein extraction

Whole brains were dissected, and HPT cells were isolated, rinsed three times with PBS and prepared for western analysis, immunoprecipitation and ELISA. Cell extracts for western blotting and immunoprecipitation were prepared by suspending the PBS-washed cells in NP-40 lysis buffer (50 mM Tris (pH 8.0), 150 mM NaCl, and 1.0% NP-40) with protease inhibitor cocktail tablets (Roche). Following incubation on ice for 30 min, non-extractable material was removed by centrifugation at 13,000 rpm for 10 min at 4°C. Cleared supernatants were used for immunoprecipitation, whereas whole homogenized cells were mixed with 1X SDS loading buffer with and without DTT, followed by western analysis. Cell extracts analyzed directly by ELISA were homogenized in bicarbonate/carbonate coating buffer (pH 9.6).

### Western blot analysis

Protein samples were separated by 12.5% SDS-PAGE and transferred to PVDF membranes (Bio-Rad, America) in electroblotting buffer (25 mM Tris, 190 mM glycine, 20% methanol) for 120 min. After rinsing with TBST buffer, the membranes were immersed in blocking buffer (5% skim milk powder in TBST) at 4°C, overnight, followed by incubation with primary antibody for 1 h (anti-GST or anti-His diluted in 5% skim milk in TBST). Subsequently, the membranes were incubated in HRP-conjugated rabbit anti-mouse IgG (GE Healthcare) for 1 h and visualized by the enhanced chemiluminescence detection system (Amersham Biosciences). The X-ray images from western blotting were analyzed according to the Quantity One user guide. Briefly, the western blotting films were scanned and saved as digital images as a quantity-one file (or .1sc) by GS-800 calibrated imaging densitometer. These quantity-one files were used for protein analysis. Protein bands in all scanned images (.1sc file) were quantified and the values of the band intensities were calculated by using the Volume and Match tools (Quantity One software version 4.6.0; Bio-Rad Laboratories). These values were used to perform statistical analysis as described in the “Statistical analysis” part below.

### Immunoprecipitation

Immunoprecipitations were performed by first incubating cell lysates from brain or HPT with the indicated primary antibodies overnight at 4°C. Immune complexes were then precipitated by incubating reactions for an additional 2 h at 4°C with either Sepharose-conjugated protein A or agarose-conjugated protein G. The immunoprecipitates were washed four times with 1% Triton X-100 lysis buffer and were resuspended in SDS-PAGE sample buffer for western blotting.

### Transcription analysis

The transcript levels of AST1 and AST2 were detected by quantitative RT-PCR using QuantiTect SYBR green PCR kit (QIAGEN). The relative expression was normalized to the expression of the mRNA encoding the crayfish ribosomal protein gene (R40s) for each sample. The primers used are shown in Table S2. The qPCR reactions contained 5 µl of 1∶10 diluted cDNA template, 1xQuantiTect SYBR Green PCR master mix (QIAGEN) and 5 µM forward and reverse primers in a 25 µl reaction volume. The following amplification profile was used: 95°C for 15 min, followed by 45 cycles of 94°C for 15 s, 58°C for 30 s, and 72°C for 30 s. All qPCR reactions were performed in triplicates. The hemocytes, HPTs and brains from a least three crayfish were used for each time point. The statistical comparisons were performed as shown below (Statistical analysis).

### ELISA

Cell extracts, containing protein at 20 µg/ml were coated in wells and incubated for 2 h at room temperature, followed by incubation with blocking solution (1% BSA in PBS). Following three careful washes with PBS, the different proteins were detected with the corresponding primary antibody (1∶1000) followed by HRP-conjugated secondary antibodies (1∶3000). After the addition of 100 µl tetramethylbenzidine (TMB) substrate (Sigma) and incubation for 20 min, the reaction was terminated by 100 µl of stop solution (0.5 M sulfuric acid) and the absorbance of the resulting color was measured at 450 nm. All samples were performed in triplicates and each experiment was repeated three times.

### Antibodies

Polyclonal antibodies against recombinant crayfish AST1 and AST2 were raised in rabbit as have been described earlier [31]. A goat polyclonal antibody to human BMAL1 (N-5: SC-8550) and goat polyclonal antibody to mouse CLK (S-19: SC-6927) were obtained from Santa Cruz Biotechnology. A goat polyclonal antibody to RACK1 (GNB2L1: Orb22484) was obtained from Biorbyt. A goat polyclonal antibody against actin (C-11: SC-1615) was used as internal control. The specificity of each antibody was tested by western blots, and all were found to be specific for each protein.

### Electrophoretic mobility shift assay (EMSA)

Mobility shift assays were performed according to reference [53]. Briefly, a synthetic fluorophore labeled oligonucleotide probe including an E-box element ( CACGTG ) was used as a substrate in this assay. To generate an E-box containing double-stranded DNA fragment, the two fluorophore labeled E-box oligonucleotides described below were annealed. A 30 µL EMSA reaction mixture contained ∼100 mM KCl, 50 ng of crude crayfish brain lysates, 1 µg poly (dI-dC), and 10 fmol of labeled probe. For control 10 fmol of unlabeled competitor oligonucleotide or mutant E-box oligonucleotide were incubated as control. After incubation for 1 hour on ice, antibodies against CLK protein was added and incubated another 20 minutes on ice. Protein-DNA complexes were resolved by 5% polyacrylamide gel electrophoresis. Specific DNA-protein and antibody-supershifted complexes were observed as retarded bands in the gel. E-box (5′-TTT AGT GAA AAG CCG CCG CTC ACG TGG CGA ACT GCG TGA CTT G-3′ and 5′-TTT CAA GTC ACG CAG TTC GCC ACG TGA GCG GCG GCT TTT CAC T-3′) and E-box mutant (5′-TTT AGT GAA AAG CCG CCG CTC AGC TGG CGA ACT GCG TGA CTT G-3′ and 5′-TTT CAA GTC ACG CAG TTC GCC AGC TGA GCG GCG GCT TTT CAC T-3′) sequences were used in the gel shift analysis (the E-box, and E-box mutant sequence is underlined).

### Statistical analysis

All statistical comparisons were examined by one-way analysis of variance, followed by Duncan's new multiple-range test and the Tukey test. When two treatments were compared, a Student's paired t-test was used. Differences were considered statistically significant at P<0.05 and/or P<0.01. The results are expressed as the mean ± standard deviation (SD).

## Supporting Information

Figure S1 A) The specific binding of AST1 and AST2 antibodies was detected by western blotting of a hemocyte lysate. B) AST2 protein was detected only inside the cell, whereas the AST1 could be detected in both plasma and cytoplasm of the hemocytes.
(TIF)

Figure S2 Amino acid sequence alignment of *Pl*RACK1 with other RACK1 sequences from other species: mouse-RACK1 (*Mus musculus*, BAE40059.1), human-RACK1 (*Homo sapiens*, BAD96208.1), Zebrafish (*Danio rerio*, NP571519.1), shrimp-RACK1 (*P. monodon*, ABU49887.1), crayfish-RACK1 (*P. leniusculus*) and fruit fly-RACK1 (*D. melanogaster*, NP477269.1). The sequences of *Pl*RACK1 were subjected to conserved domain analysis at NCBI to predict the presence of the WD40 repeats. Positions of the seven WD repeats (WD1–7) are indicated with arrows.
(TIF)

Figure S3 *Pl*RACK1 is expressed in all tested tissues in *P. leniusculus*. The experimental tissues examined included muscle (M), hemocytes (HC), heart (HE), gill (G), hepatopancreas (HP), hematopoietic tissue (HPT), abdominal nerve (N), eyestalk (ES), intestine (IN), testis (TT), and brain (B). A 40S ribosomal gene was used as internal control.
(TIF)

Figure S4 A) Schematic representation of the alignment in BMAL1 proteins. Full-length amino acid sequences and conserved domains of BMAL1 from three organisms were aligned. Overall % identity is shown. The black boxes represent the conserved domains and % identities of these domains. B) RT-PCR analysis of *Pl*BMAL1 in different crayfish tissues, consisting of hemocytes (HC), hepatopancreas (HP), testis (TT), heart (HE), intestine (IN), gill (G), abdominal nerve (N), muscle (M), eyestalk (ES), brain (B), and hematopoietic tissue (HPT). The 40S ribosomal gene was used as the internal control in all tissues.
(TIF)

Figure S5 The expression and purification of GST-*Pl*RACK1, His-Trx-AST2, and tag proteins. A) The GST-*Pl*RACK1 was analyzed by 12.5% SDS-PAGE. Lane M is protein molecular weight markers; lane 1 and 2 show the expression of the GST-*Pl*RACK1 before and after induction; lane 3 is the soluble fraction and lane 4 is the insoluble pellet of the cell lysate; lane 5 is the purified- GST-*Pl*RACK1 protein from the column after dissolution of the inclusion bodies and refolding. B) The expressed proteins: GST, thioredoxin and His-Trx-AST2 were analyzed by 12.5% SDS-PAGE. Lane M is protein molecular weight markers; lane 1 and 2 show the expression of proteins before and after induction; lane 3 shows the purified proteins.
(TIF)

Figure S6 The expression of recombinant *Pl*BMAL1 in *E.coli.* A) Recombinant His-Trx-*Pl*BMAL1 was analyzed by 10% SDS-PAGE, and B) western blot. Lane M, protein molecular weight markers; lane 1 and 2 show expression of recombinant protein before and after induction; lane 3 and 4 show the protein from supernatant and insoluble pellet of the cell lysate respectively; lane 5 shows the purified His-Trx-*Pl*BMAL1. C) Recombinant GST-*Pl*BMAL1 was analyzed by 10% SDS-PAGE. Lane M, protein molecular weight markers; lane 1–3 show the expression of the GST-*Pl*BMAL1 at 0 h, 4 h and overnight respectively; lane 4–5 show the soluble fraction and insoluble pellet of the cell lysate; lane 6 shows the purified-GST-*Pl*BMAL1 protein.
(TIF)

Figure S7 AST2 can't bind to BMAL1 directly. *In vitro* GST pull-down assay of His-Trx-*Pl*BMAL1 by GST-AST2, the eluted fractions were examined by western blotting using anti-GST or anti-His antibodies. The recombinant GST was used as internal control.
(TIF)

Figure S8 A) Crayfish were treated with dsGFP or dsAST2, and then crude brain lysates were harvested during day and night, and used in EMSA assay. The E-box binding activity of CLK-*Pl*BMAL1 is indicated on the right side of the gel. A competitive binding with unlabeled E-box was used as a control. The horizontal band on top of the gel indicates day (white) or night (black). B) The crayfish were injected with melatonin or crayfish saline as control, during daytime. At 3 h post injection, the DNA binding activities of brain lysates were analyzed by EMSA (lane 1 and 2). A supershift EMSA using preincubation of the lysate with anti-CLK Ab (lane 3 and 4) or competitive binding with unlabeled E-box (lane 5 and 6) were also performed. The CLK-*Pl*BMAL1 specific mobility shift is indicated on the right side of the gel. C) The presence of CLK-*Pl*BMAL1 proteins in the specific shift bands were confirmed by cutting the bands and homogenizing in SDS-PAGE buffer followed by detection by western blot using antibodies against CLK and BMAL1 respectively.
(TIF)

Table S1 Mascot search result for protein detected as AST2-binding in a GST pull-down and far overlay assay. Ions score is −10*Log(P), where P is the probability that the observed match is a random event. Individual ions scores >61 indicate identity or extensive homology (p<0.05). Protein scores are derived from ions scores as a non-probabilistic basis for ranking protein hits. A protein score >70 is considered as significant (p<0.05).
(DOCX)

Table S2 Sequences of the primers used in this study.
(DOC)
